The article "Astaxanthin Prevents Tuberculosis-Associated Inflammatory Injury by Inhibiting the Caspase 4/11-Gasdermin-Pyroptosis Pathway" was published in 2022. Journal: Evid Based Complement Alternat Med.

# Astaxanthin Prevents Tuberculosis-Associated Inflammatory Injury by Inhibiting the Caspase 4/11-Gasdermin-Pyroptosis Pathway

**DOI:** 10.1155/2022/4778976

**Published:** 2022-12-06

**Authors:** Li Li, Zulipikaer Abudureheman, Xuemei Zhong, Liang Gao, Hui Gong, Chuanjiang He, Boyi Yang, Jie Ren, Ayiguli Alimu, Subinuer Yilamujiang, Fan Yang, Xiaoguang Zou

**Affiliations:** ^1^Department of Respiratory and Critical Care Medicine, First People's Hospital of Kashi, Kashi, China; ^2^State Key Laboratory of Pathogenesis, Prevention and Treatment of High Incidence Diseases in Central Asia, Xinjiang Medical University, Urumqi, China; ^3^Department of Clinical Research Center of Infectious Diseases (Pulmonary Tuberculosis), First People's Hospital of Kashi, Kashi, China; ^4^Department of Clinical Laboratory, First People's Hospital of Kashi, Kashi, China; ^5^Department of Preventive Medicine, Sun Yat-Sen University, Guangzhou, China; ^6^Department of Infectious Disease, First People's Hospital of Kashi, Kashi, China

## Abstract

Pyroptosis is a programmed cell death caused by inflammation. Multiple studies have suggested that Mycobacterium tuberculosis infection causes tissue pyroptosis. However, there are currently no protective drugs against the inflammatory damage caused by pyroptosis. In this study, anti-pyroptotic effects of the natural compound astaxanthin (ASTA) were explored in a simulated pulmonary tuberculosis-associated inflammatory environment. The results showed that ASTA maintained the stability of MLE-12 lung epithelial cell numbers in the inflammatory environment established by lipopolysaccharide. The reason is not to promote cell proliferation but to inhibit lipopolysaccharide-induced pyroptosis. The results showed that ASTA significantly inhibited the expression of key proteins in the caspase 4/11-gasdermin D pathway and the release of pyroptosis-related inflammatory mediators. Therefore, ASTA inhibits inflammation-induced pyroptosis by inhibiting the caspase 4/11-gasdermin D pathway and has the potential to protect lung tissue from tuberculosis-related inflammatory injury. ASTA, a functional food component, is a promising candidate for protection against tuberculosis-associated inflammatory lung injury.

## 1. Introduction

Tuberculosis (TB) remains a leading cause of infectious death worldwide [1]. Pulmonary tuberculosis has obvious symptoms such as cough, sputum, and hemoptysis [2]. This is closely related to the lung damage caused by TB. TB presents as “latent” TB and “active” TB disease, and the treatment for each is different [3]. Isoniazid is excellent for the former, and rifampin is excellent for the latter. Pyrazinamide and ethambutol complete the first-line regimen for drug-susceptible TB, each playing a specific role [4, 5]. At present, the inhibitory therapy against Mycobacterium tuberculosis (MTB) has achieved good results, but inflammatory lung injury caused by TB is a key factor, affecting the quality of life of patients [6]. Importantly, the factors causing lung impairment remain unclear. Host immune responses probably play a dominant role in lung damage, as excessive inflammation and elevated expression of lung matrix-degrading proteases are common during TB [7]. According to reports, MTB can cause pyroptosis through multiple pathways leading to inflammation or inflammatory damage [8–10]. TB causes caspase-1/NLRP3/gasdermin D-mediated pyroptosis of human monocytes and macrophages [8].

Pyroptosis, also known as inflammatory necrosis, is a type of programmed cell death, which is characterized by the continuous expansion of cells until the cell membrane ruptures, resulting in the release of cell contents and the activation of a strong inflammatory response [11]. Pyroptosis is an important innate immune response in the body and plays an important role in fighting infections [12]. Several studies have confirmed that pyroptosis is an important cause of lung injury in the process of pulmonary inflammatory diseases [13, 14]. Therefore, regulation of pyroptosis may be the strategy to protect against TB-related inflammatory lung injury.

Natural compounds can be used as references for drug development [15–17]. Astaxanthin (ASTA) is a keto carotenoid whose chemical name is 3, 3′-dihydroxy-4, 4′-diketo-*β*, *β*′-carotene. It is widely found in shrimps, crabs, fish, birds, some algae, fungi, and other organisms [18]. The antioxidant and immune-promoting effects of astaxanthin can be used to prevent oxidative tissue damage [19]. However, studies on its regulatory role in inflammation are limited. In a previous study, we confirmed that astaxanthin can effectively reduce lipopolysaccharide (LPS)-induced apoptosis. Based on the previous studies, this study explores the effect of ASTA on lung injury caused by TB-related inflammation based on the pyroptotic pathway.

## 2. Materials and Methods

### 2.1. Chemicals and Reagents

ASTA and disulfiram (TETD) were obtained from MedChemExpress (New Jersey, USA). The purity of these compounds was >95%. ECL chemiluminescence kit, DAPI fluoromount-GTM mounting medium, cell counting kit-8 (CCK-8), and dimethyl sulfoxide (DMSO) were obtained from YEASEN (Shanghai, China). Hoechst 33342 was purchased from Solarbio (Beijing, China). Fetal bovine serum (FBS) was obtained from ExCell Bio (Shanghai, China). RPMI medium modified (1640) was obtained from Hyclone, Thermo Scientific (MA, USA). A cell cycle staining kit was provided by Multi Sciences (Hangzhou, China). Antibodies against caspase 4, caspase 11, gasdermin D, GAPDH, and HRP-labeled goat antirabbit IgG (H + L) were obtained from Immunoway (Plano, TX, USA). Antibodies against cyclin A2 (CCNA2), cyclin B1 (CCNB1), and cyclin E1 (CCNE1) were purchased from HUABIO (Hangzhou, China).

### 2.2. Cell Culture

The mouse alveolar epithelial cell line MLE-12 was obtained from OTWO Biotech INC (Shenzhen, China) and maintained at 37°C under 5% CO_2_ in an RPMI 1640 medium (Hyclone, MA, USA) supplemented with 10% FBS (ExCell Bio, Shanghai, China).

### 2.3. Coculture

MLE-12 cells were seeded in a 12-well plate (1 × 10^4^ cells/well) (Corning Incorporated, Corning, MA) and cultured overnight. RWA264.7 macrophages were added at a ratio of 1 : 1 with a fresh medium grown for 4 h. LPS or ASTA was added to the medium and grown for 24 h at 37°C under 5% CO_2_. The nuclei were marked with the Hoechst 33342 stain (Solarbio, Beijing, China). Changes in the morphology and cell membrane of the MLE-12 cells were observed using a high content analysis system (PerkinElmer, Operetta CLS).

### 2.4. Dynamic Cell Morphology Monitoring

Real-time cell morphology was monitored using a high content analysis system (PerkinElmer, Operetta CLS). MLE-12 cells were seeded in a 96-well plate (1 × 10^3^ cells/well) (Corning Incorporated, Corning, MA) and cultured overnight with different compounds. The shape of cells was dynamically monitored by using the content analyzer for 24 h. All experiments were independently repeated three times.

### 2.5. Cell Viability Assay

The inhibitory effect of ASTA on the viability of the MLE-12 cells was measured with the CCK-8 assay. In brief, the cells were seeded in 96-well plates (Corning Incorporated, Corning, MA) at a density of 5 × 10^3^ cells/well in 200 *μ*L of the culture medium and grown for 4 h at 37°C under 5% CO_2_. Next, they were treated with different concentrations of ASTA for 24 h. Subsequently, 10 *μ*L of CCK-8 solution was added to each well, and the plates were incubated for 1 h at 37°C in a 5% CO_2_ atmosphere. The optical density of each well was determined at 450 nm using a microplate reader (Bio-Rad, Hercules, CA). All experiments were independently repeated three times.

### 2.6. Cell Cycle Analysis

MLE-12 cells in the logarithmic growth phase were seeded in a 6-wellflat-bottom plate at the standard of 2 mL cell suspension at 24 h. The cell suspensions were centrifuged at 181 × *g* for 5 min, and after that, the cell pellets were collected. After using chilled PBS to wash twice, 600 *µ*L of DNA staining solution and 10 *µ*L of permeabilization buffer (Multi Sciences, Hangzhou, China) were added. After incubation in the dark for 30 min at 4°C, flow cytometric analysis was performed. All experiments were independently repeated three times.

### 2.7. Western Blot Analysis

MLE-12 cells were cultured overnight in six-well plates (1 × 10^5^ cells/well) and treated with LPS and other compounds. Protein lysates were separated using sodium dodecyl sulfate-polyacrylamide gel electrophoresis and transferred into nitrocellulose membranes. The membranes were blocked at room temperature for 2 h with 5% skim milk in tris-buffered saline/tween 20 and then incubated overnight at 4°C with primary antibody specifics for CCNA2, CCNB1, CCNE1, caspase 4, caspase 11, and gasdermin D. Goat antirabbit IgG was used as a secondary antibody to incubate the membranes at room temperature for 2 h. The bands formed were visualized using the enhanced chemiluminescence detection system (BioRad ChemiDocTM XRS+), and specific signals were quantified using densitometric analysis (Image J software). All experiments were independently repeated three times.

### 2.8. Enzyme-Linked Immunosorbent Assay

The cell supernatants were collected after centrifugation. Next, IL-1*β*, IL-18, and LDHA contents of the supernatants were assayed using the enzyme-linked immunosorbent assay (ELISA) according to the manufacturer's protocol (Cayman Chemicals, Ann Arbor, MI, USA). The optical density of each well was determined using a microplate reader (Bio-Rad, Hercules, CA). All experiments were independently repeated three times.

### 2.9. Statistical Analysis

Analyses were performed using SPSS version 24.0 (USA). The results are presented as a mean ± standard deviation (SD) of at least three independent experiments. One-way analysis of variance (ANOVA) and Student's *t*-test were used to compare groups. *∗P*  <  0.05 was considered significant.

## 3. Results

### 3.1. ASTA Maintains the Stable Number of MEL-12 Cells

From previous experiments, we found that 15 *μ*mol/L is the minimum concentration of ASTA to promote the proliferation of MEL-12 cells and that 8 *μ*g/L is the minimum concentration to inhibit the proliferation of MEL-12 cells. Therefore, we used 8 *μ*g/L LPS to establish a pulmonary tuberculosis-related alveolar epithelial cell inflammatory injury model and then intervened MEL-12 cells with 15 *μ*mol/L ASTA.

In this study, we first examined the experimental concentration of TETD. As shown in Figure 1(a), when the TETD concentration was higher than 7.5 *μ*mol/L and cells were incubated for 24 h, cell proliferation decreased. Therefore, we determined the experimental concentration of TETD to be 7.5 *μ*mol/L. To evaluate the effects of ASTA on MLE-12 cells with LPS, a high content analysis system was used to monitor the cell numbers. As shown in Figure 1(b), LPS inhibits the number of MLE-12 cells, whereas both ASTA and TETD maintain the stable number of MEL-12 cells.

### 3.2. ASTA Does Not Affect Cell Proliferation Inhibition by LPS

The results show that ASTA prevented LPS-induced cell number reductions. We believe that this result may be due to two reasons: one is that ASTA promotes cell proliferation and the other is that ASTA prevents LPS-induced cell death. We first observed the effect of ASTA on MEL-12 cell proliferation in an inflammatory environment. We examined the effect of ASTA on the cell cycle using flow cytometry. As shown in Figure 2(a), LPS induced a significant decrease in both the S phase and G2 phase of the MLE-12 cell cycle, suggesting that cell proliferation was inhibited. However, ASTA did not improve the inhibition of cell proliferation caused by LPS. We further detected the expression of cyclins CCNA2, CCNB1, and CCNE1 using western blotting and found the same change in the trend in the cell cycle (Figure 2(b)).

### 3.3. ASTA Inhibits MLE-12 Cell Pyroptosis

We found that ASTA did not change the LPS-induced inhibition of MLE-12 cell proliferation. Therefore, the reason why ASTA maintained the stability of the cell number is most likely that it inhibited LPS-induced cell death. We confirmed in another study that ASTA can inhibit LPS-induced apoptosis of MLE-12 cells. However, some reports suggest that associated pulmonary inflammatory injury may also be closely related to the pyroptosis of alveolar epithelial cells [20, 21]. In addition, we also observed in the above experiments that the pyroptosis inhibitor TETD maintained the stability of the number of MLE-12 cells in the inflammatory environment. It is suggested that LPS caused the pyroptosis of MLE-12 cells, and the number of MLE-12 cells was maintained after the inhibition of pyroptosis. Based on the above analysis, we further observed whether ASTA plays any role in LPS-induced pyroptosis through dynamic observation.

Macrophages are the key inflammatory cells in inflammation-induced pyroptosis [22]. Many inflammatory factors secreted by macrophages can cause tissue cell pyroptosis. To observe more directly whether LPS induces inflammatory cell aggregation and induces pyroptosis of alveolar epithelial cells, we established a coculture system of alveolar epithelial cells and macrophages. As shown in Figure 3, through dynamic observation, we found that LPS induced obvious changes in cell morphology––cells increasingly swell, cell membranes rupture, and cells die. However, the cell morphology in the ASTA and TETD groups did not change significantly after 24 h. Through this phenomenon, we preliminarily confirmed the speculation that ASTA can inhibit the pyroptosis of MLE-12 cells.

### 3.4. ASTA Inhibits the Caspase 4/11-Gasdermin D Pyroptosis Pathway

LPS usually induces pyroptosis through the nonclassical pathways. LPS does not directly enter the cytoplasm through receptors. Other caspase family members such as caspase 4, 5, and 11 are activated [23, 24]. The activated caspases 4, 5, and 11 cleave to gasdermin D and induce pyroptosis [25]. Therefore, we detected the expression of key proteins caspase 4, caspase 11, and gasdermin D in the pyroptosis pathway using western blotting. LPS significantly induced increased expression of caspase 4, caspase 11, and gasdermin D. ASTA reversed the changes in the levels of these proteins. TETD also significantly reduced the expression of gasdermin D (Figures 4(a) and 4(b)). The above experiments suggest that ASTA inhibits LPS-induced pyroptosis of MLE-12 cells by inhibiting the caspase 4/11-gasdermin D pathway.

### 3.5. ASTA Reduces Pyroptosis-Related Inflammatory Mediator Release

In addition to the direct induction of pyroptosis by LPS, IL-1*β*, IL-18, and LDHA produced by pyroptosis will further expand the inflammatory response and cause significant inflammatory damage [26, 27]. Using the ELISA, we found that ASTA and TETD significantly reduced the release of inflammatory mediators such as IL-1, IL-18, and LDHA (Figures 5(a)–5(c)).

## 4. Discussion

In another study, we focused on the protective effects of ASTA on TB-related inflammatory injury, which was mainly explained by the apoptotic pathway. In our further literature study, we found that pyroptosis is also an important mechanism that causes pulmonary inflammatory damage. Therefore, based on the previous discovery that ASTA has an inhibitory effect on inflammatory damage, we further explored whether it also acts through the pyroptosis pathway. Pyroptosis, also known as cell inflammatory necrosis, is a type of programmed cell death. Pyroptosis is a new type of programmed cell death discovered and confirmed in recent years, which is characterized by its dependence on inflammatory caspases (mainly caspase 1, 4, 5, and 11) and accompanied with the release of many proinflammatory factors [23–25]. The morphological characteristics, occurrence, and regulatory mechanisms of pyroptosis are different from other cell death methods such as apoptosis and necrosis. Research shows that pyroptosis is widely involved in infectious diseases [28].

First, we found that both ASTA and the pyroptosis inhibitor TETD, which target gasdermin D, maintained stable MLE-12 cell numbers in an LPS-mimicking inflammatory environment. It may be due to two reasons: one is that ASTA and TETD promote cell proliferation and the other is that ASTA prevents LPS-induced cell death. Therefore, we further analyzed the effect of ASTA and TETD on the proliferation of MLE-12 by detecting the cell cycle. The results show that ASTA did not promote MEL-12 cell proliferation in an inflammatory environment. This suggests that ASTA maintains stable MLE-12 cell numbers in an inflammatory environment by reducing cell death.

We found that the pyroptosis inhibitor TETD could also maintain the stability of MLE-12 cell numbers in the LPS-induced inflammatory microenvironment. This provided a basis for our further exploration of the aspect of scorching death. Pyroptosis manifests as cell swelling and cell membrane rupture. In the established coculture system of MEL-12 cells and RAW246.7 macrophages, we found that LPS could significantly cause cell swelling and cell membrane rupture. However, the morphology of MLE-12 cells did not change much after ASTA and TETD intervention. The above results suggest that LPS induced pyroptosis in MLE-12 cells. Cell numbers can be stabilized by preventing pyroptosis. ASTA also inhibits pyroptosis. In the noncanonical pathway, caspase 4/11 can be activated through direct contact with bacterial LPS and then cleaved to gasdermin D, triggering pyroptosis. Next, we further investigated the anti-pyroptotic mechanisms of ASTA. We found that ASTA can inhibit the activation of the caspase 4/11-gasdermin D pathway. In addition, ASTA also significantly inhibited the production of pyroptosis-related inflammatory mediators.

## 5. Conclusion

Based on the previous confirmation that ASTA can reduce LPS-induced MLE-12 cell apoptosis, we also confirmed in this study that ASTA can also inhibit LPS-induced pyroptosis through the caspase 4/11-gasdermin D pathway (Figure 6). Therefore, we are more convinced that ASTA is a natural compound worthy of attention and development in the treatment of pulmonary tuberculosis.

## Figures and Tables

**Figure 1:** ASTA maintains MLE-12 cell survival. (a) CCK-8 assay shows the viability rate of the MLE-12 cells after different concentrations of ASTA treatments. (b) Real-time monitoring of unlabeled MLE-12 cell survival within 24 h. The data are presented as a mean ± SD.  ^*∗*^*P*  <  0.05 compared with the control.

**Figure 2:** ASTA did not significantly change the period field of the MLE-12 cells induced by LPS. (a) Cell cycle after different treatments using flow cytometry. (b) Western blotting shows the protein expression of CCNA2, CCNB1, CCNE1, procaspase 3, and caspase 3 in MLE-12 cells. The data are presented as a mean ± SD.  ^*∗*^*P*  <  0.05,  ^*∗∗*^*P* <  0.01 compared with the control.

**Figure 3:** ASTA inhibits MLE-12 cell pyroptosis. Morphological changes by pyroptosis were observed using laser confocal microscopy. The yellow arrows mark the cell membrane of MLE-12 cells.

**Figure 4:** ASTA inhibits pyroptosis of MLE-12 cells by inhibiting the caspase 4/11-gasdermin D signal pathway. (a, b) Western blotting and immunofluorescence showing the protein levels of caspase 4, caspase 11, and gasdermin D in MLE-12 cells. The data are presented as a mean ± SD.  ^*∗*^*P*  <  0.05,  ^*∗∗*^*P*  <  0.01 compared with the control.

**Figure 5:** ASTA inhibits MLE-12 cell pyroptosis-related cytokine release. (a)–(c) IL-1*β*, IL-18, and LDHA content of MLE-12 cells.

**Figure 6:** The mechanisms of action of ASTA.

## Data Availability

The data used to support the findings of this study are available from the corresponding author upon request.
